The article "Silencing of BAG3 inhibits the epithelial-mesenchymal transition in human cervical cancer" was retracted in 2025. Reasons: plagiarized images; overlap with other authors' work; concerns about the results or conclusions.

# Silencing of BAG3 inhibits the epithelial-mesenchymal transition in human cervical cancer

**DOI:** 10.18632/oncotarget.20726

**Published:** 2017-09-08

**Authors:** Fei Song, Geng Wang, Zhifang Ma, Yuebing Ma, Yingying Wang

**Affiliations:** ^1^ Department of General Surgery, Shandong Provincial Third Hospital, Jinan, Shandong, China; ^2^ Department of Emergency, Laiwu City People's Hospital, Laiwu, Shandong, China; ^3^ Department of Gynecologic Oncology, Shandong Cancer Hospital Affiliated to Shandong University, Shandong Academy of Medical Sciences, Jinan, Shandong, China

**Keywords:** BAG3, EMT, cervical cancer

## Abstract

Bcl2-associated athanogene 3 (BAG3) has been reported to be involved in aggressive progression of many tumors. In the present study, we examined the expression of BAG3 in human cervical cancer (CC) tissues and investigated the role of BAG3 in SiHa and HeLa cell growth, migration, and invasion. Here, we found that most of CC tissues highly expressed the protein and mRNA of BAG3, while their expression was obviously lower in paired normal tissues (all p<0.001). BAG3 expression was associated with FIGO stage and metastasis (all p<0.05). *In-vitro* analysis demonstrated that BAG3 siRNAs inhibited SiHa and HeLa cell growth, invasion and migration. Mechanically, BAG3 siRNAs inhibited the expression of EMT-regulating markers, involving MMP2, Slug and N-cadherin, and increased the expression of E-cadherin. In a xenograft nude model, BAG3 siRNAs inhibited tumor growth and the expression of EMT biomarkers. In conclusion, BAG3 is involved in the EMT process, including cell growth, invasion and migration in the development of CC. Thus, BAG3 target might be recommended as a novel therapeutic approach.

## INTRODUCTION

To data, cervical cancer has been reported to be the second most common cancers in the department of gynecology [1]. Most of cervical cancer patients, especially patients with International Federation of Gynecology and Obstetrics (FIGO) IB2 stage, will develop the recurrence and distant metastasis [2]. As reported, various genes and proteins, such as the high mobility group box l [3], metastasis-associated 1 [4], Twist [5], were demonstrated to be related to the development of cervical cancer. Thus, it is important to understand the mechanisms underlying cancer cell invasiveness and metastasis.

BAG3, a member of six BAG families, contains a conserved domain, and interacts with Hsp-70 [6–9]. It has been reported that BAG3 is highly expressed in many kinds of primary tumors, including ovarian cancer, and glioblastoma [10–13]. In addition, BAG3 is able to modulate some tumor biology processes, involving cell apoptosis, growth, cytoskeleton organization, and differentiation [14, 15]. Some studies have reported that the overexpression of BAG3 inhibits drug-induced or serum-deprivation apoptosis in some degree and the inhibition of BAG3 promotes tumor cell apoptosis. What is more, BAG3 was reported to be involved in the angiogenesis in endothelial cells via ERK phosphorylation [16]. However, little is known about the role of BAG3 in cervical cancer.

The article "Silencing of BAG3 inhibits the epithelial-mesenchymal transition in human cervical cancer" was retracted in 2025. Reasons: plagiarized images; overlap with other authors' work; concerns about the results or conclusions.

In the present study, we examined the expression of BAG3 in human cervical cancer tissues and investigated the role of BAG3 in SiHa and HeLa cell growth, migration, and invasion. This study provides evidence that BAG3 can increase the EMT nature in cervical cancer cells.

## RESULTS

### Expression of BAG3 in cervical cancer tissues and cells

To explore the BAG3-EMT signaling pathway in the development of human cervical cancer, we used RT-PCR and immunoblotting to investigate the expression of BAG3 in 30 cases of cervical cancer tissues. As illustrated in Figure 1, RT-PCR assay showed that the expression intensity of BAG3 in cervical cancer tissues was 1.21±0.12. However, BAG3 mRNA was rarely expressed in paired normal samples with the expression intensity 0.12±0.03 (Figure 1a). In addition, immunoblotting revealed that the expression intensity of BAG3 protein in all cervical cancer tissues was 1.13±0.13, However, BAG3 protein was rarely expressed in surrounding non-tumor samples with expression intensity 0.15±0.04 (Figure 1b). At the same time, the expression of BAG3 was further detected in HeLa and SiHa cell lines using RT-PCR and immunoblotting. We found that BAG3 mRNA and protein were highly expressed in HeLa and SiHa cell lines than NEEC cells (Figure 1c, 1d). These results indicate that BAG3 was involved into the development of human cervical cancer.

**Figure 1:** Expression of BAG3 in cervical cancer tissues and cells **(a)** RT-PCR analysis demonstrates that BAG3 expression was significantly suppressed in cancer tissues compared with normal tissues. **(b)** RT-PCR analysis demonstrates that BAG3 expression was significantly suppressed in HeLa and SiHa cells compared with normal NEEC cells. **(c)** Western blot analysis demonstrates that BAG3 expression was significantly suppressed in cancer tissues compared with normal tissues. **(d)** Western blot analysis demonstrates that BAG3 expression was significantly suppressed in HeLa and SiHa cells compared with normal NEEC cells. GAPDH primers and antibody were used as an equal loading control.

### Correlations between BAG3 and clinicopathology

Based on results above, we analyzed the association of BAG3 expression with clinicopathological parameters in cervical cancer. As shown Table 1, the expression of BAG3 mRNA was obviously increased in patients with advanced FIGO IB2 stage than those in early FIGO stage (p=0.006). In addition, the expression of BAG3 mRNA was closely positively correlated with lymph node metastasis (p=0.006). However, no discernible associations were observed in age, tumor size and differentiation. Besides, the expression of BAG3 protein was also obviously increased in advanced FIGO IB2 stage those in early FIGO stage (p=0.043). At the same time, the expression of BAG3 protein was closely positively correlated with lymph node metastasis (p=0.016). However, age, tumor size and differentiation showed no associations with BAG3 protein.

The article "Silencing of BAG3 inhibits the epithelial-mesenchymal transition in human cervical cancer" was retracted in 2025. Reasons: plagiarized images; overlap with other authors' work; concerns about the results or conclusions.

**Table 1:** BAG3 expression in cervical cancer according to clinicopathologic characteristics

Variables	Number	mRNA	P value	Protein	P value
Age					
<41	15	1.19±0.13	0.388	1.09±0.15	0.699
≥41	15	1.23±0.12		1.11±0.13	
FIGO stage					
IB2	12	1.13±0.13	0.006	1.06±0.12	0.043
>IB2	18	1.28±0.14		1.15±0.11	
Size of tumor (cm)					
<4	16	1.17±0.15	0.414	1.08±0.13	0.424
≥4	14	1.22±0.18		1.12±0.14	
Differentiation					
Grade 1/2	13	1.16±0.21	0.205	1.08±0.14	0.379
Grade 3	17	1.25±0.17		1.13±0.16	
LN Metastasis					
Yes	15	1.31±0.21	0.006	1.21±0.16	0.016
No	15	1.09±0.19		1.05±0.18	

### BAG3 siRNAs inhibit cell growth of HeLa and SiHa cells

To explore the effect of BAG3 on a series of biological processes of HeLa and SiHa cells, BAG3 siRNAs (si-BAG3) were utilized to knock down the endogenous BAG3 expression. After transfection, RT-PCR and western blotting analysis verified that the expression of BAG3 protein in HeLa and SiHa cells transfected with BAG3 siRNAs was obviously reduced (Figure 2a). Next, HeLa and SiHa cell growth following BAG3 siRNAs were examined using cell proliferation assay, and cells with the empty vector were used as control (Figure 2b). We found that BAG3 siRNAs inhibited HeLa and SiHa cell growth rate within 72 hours with significant significances (p<0.001, p<0.001, respectively).

**Figure 2:** Effect of knock-down of BAG3 on cell growth of CC cell lines **(a)** RT-PCR (28 cycles) showed decreased BAG3 mRNA transcripts in the si-BAG3-transfected cells compared to controls (si-control) in HeLa and SiHa cells. GAPDH (25 cycles) was examined as an equal loading control. Knock-down of BAG3 protein in the same cells was verified by Western blot analysis. GAPDH antibody was used as the loading control. **(b)** Cell numbers were measured by crystal violet absorbance after 1, 2 and 3 days growth and results expressed as % cell number on day 2 and 3 compared to day 1. After 3 days, growth was decreased in comparison with the controls. Data was analysed by paired t-test.^*^ indicates p<0.01. The error bars represent mean ± SD, data shown is mean of three independent experiments.

The article "Silencing of BAG3 inhibits the epithelial-mesenchymal transition in human cervical cancer" was retracted in 2025. Reasons: plagiarized images; overlap with other authors' work; concerns about the results or conclusions.

### BAG3 siRNAs inhibit HeLa and SiHa cell migration

In the present study, we used the wounding assay to investigate the migration status of HeLa and SiHa cells. Our analysis revealed that BAG3 siRNAs caused a marked decrease in HeLa cell migration as compared with si-control (p<0.001, p<0.001, respectively) (Figure 3a, 3c). In addition, we also demonstrated that reduced BAG3 expression inhibited SiHa cell migration in comparison with si-control by measuring the wound width using the ECIS system (p<0.001, p<0.001, respectively) (Figure 3b, 3d).

**Figure 3:** Effect of BAG3 expression on migration of HeLa and SiHa cells **(a, b)** Confluent monolayers of HeLa and SiHa cells were scratched and the distance moved by cells to cover the wound was measured after 24h and compared to time 0. Photographs shown are taken at 0 and 24h are from representative experiment. The data shown is from 3 independent experiments. (**c, d)** ECIS confirmed the decreased migratory capability of HeLa and SiHa cells with knockdown of BAG3 protein expression compared to the appropriate control cells. Data show relative change in resistance from 0-10 h for each cell line and are mean of 3 independent experiments ±SD. ^*^indicates p<0.001 comparing control cells.

### BAG3 siRNAs inhibit HeLa and SiHa cell invasion

To figure out the role of BAG3 in HeLa and SiHa cell invasion, we further investigated the biological role of BAG3 siRNAs using *in vitro* invasion assays by counting cell number of the artificial basement membrane, Matrigel. We found that reduced BAG3 expression in HeLa and SiHa cells caused an approximately 50% decrease (p<0.001, p<0.001, respectively) in cell number of basal member as compared with si-control (Figure 4a).

**Figure 4:** Effect of BAG3 on the invasion of CC cells **(a)** Cell invasion through matrigel coated barrier was quantitated after fixing and staining invaded cells. Invasion capability was decreased in HeLa and SiHa cells with knockdown of BAG3 protein expression. 4 fields of view/inserts were photographed and counted. Images shown are from a typical field of view (x4 magnification). Data shown is mean ±SD cell number/membrane from 3 independent experiments. T-test compared with the controls for each cell line. ^*^ indicates p<0.001. **(b)** knockdown of BAG3 can enhance the E-cadherin expression and repress the expression of MMP2, Slug, and N-cadherin as determined by Western blot. Quantification was normalized to GAPDH. GAPDH protein was used as an internal control.

### BAG3 regulates EMT process of HeLa and SiHa

It has been reported that EMT plays an essential role in the progression of CC. In view of important functions of BAG3 in the biology of HeLa and SiHa cells, we assumed that BAG3 was involved in the EMT of cervcal cancer. Next, we detected the BAG3-related downstream molecules and EMT biomarkers using HeLa and SiHa cells and western blotting. As shown in Figure 4b, BAG3 siRNAs inhibited the expression of Slug, N-cadherin, MMP2, and promoted the expression of E-cadherin in HeLa and SiHa cells compared with si-control.

The article "Silencing of BAG3 inhibits the epithelial-mesenchymal transition in human cervical cancer" was retracted in 2025. Reasons: plagiarized images; overlap with other authors' work; concerns about the results or conclusions.

### BAG3 siRNAs suppress HeLa and SiHa cell growth in nude mice

Finally, we investigated the effect of BAG3 siRNAs on HeLa and SiHa cell growth in nude mice. In this work, HeLa and SiHa cells infected with si-BAG3 or si-control were injected subcutaneously in the dorsal parts of each nude mouse. Compared with si-control, silencing of BAG3 significantly suppressed HeLa and SiHa cell growth in nude mouse (Figure 5a). As expected, western blotting analysis from tumor masses of nude mice also demonstrated that BAG3 si-RNAs decreased the expression of BAG3, Slug, N-cadherin, and MMP2, and increased expression of E-cadherin (Figure 5b).

**Figure 5:** Knockdown of BAG3 suppresses HeLa and SiHa cell growth in nude mice **(a)** HeLa and SiHa cells stably infected with BAG3 siRNA or control siRNA cells were injected into nude mice. At the indicated times, tumors were measured with Vernier calipers (mean ± SD; n=5). ^*^p<0.01 versus corresponding control siRNA. **(b)** Immunoblot analysis of representative excised tumor from (a).

## DISCUSSION

As known to all, cervical cancer was characterized by aggressive cancer cell proliferation, migration, invasion and vascularization. Distant organ metastasis and lymph node invasion are a key process in the malignant progression of cervical cancer. In spite of great efforts on anti-cervical cancer therapy in the past decades, the five-year survival rates for cervical cancer patients are still unsatisfied, and effective drugs for the treatment of cervical cancer patients are lacking. Thus, it is essential to identify the key molecular regulators in tumourigenesis and elucidate the key signaling pathways.

BAG3 was reported to be constitutively expressed in a few of normal cell types, such as skeletal muscle cells and cardiac myocytes. BAG3 expression can be induced by surrounding stress and inflammation in some kinds of cells [17]. Notably, BAG3 is also constitutively expressed in many kinds of primary tumour tissues and cell lines, which plays an important role in the cell survival, migration and invasion via distant molecular mechanisms [15]. The present study identified that BAG3 was highly expressed in CC tissues and cell lines. Consistently, previous reports also demonstrated that BAG3 was over-expressed in colorectal and prostate cancer [10–13]. These findings indicate that BAG3 acts as an oncogene, which was responsible for the progression of cervical cancer.

The article "Silencing of BAG3 inhibits the epithelial-mesenchymal transition in human cervical cancer" was retracted in 2025. Reasons: plagiarized images; overlap with other authors' work; concerns about the results or conclusions.

The epithelial mesenchymal transition plays an important role in the migration, invasion and metastasis of cancers. In addition, it is the EMT that affects progression-free survival and overall survival of the patients [18, 19]. A large number of EMT-related molecular biomarkers and signaling have been identified. In the EMT progression, EMT features as a series of biological events, including the decreased expression of the epithelial marker E-cadherin, resulting in a lost connection between epithelial cells and decreased polarity of the epithelial cells. However, the expression of N-cadherin and Vimentin is increased, which exhibits some mesenchymal cell properties, and promotes cell migration and invasion [20]. The EMT process is modulated by a series of transcription factors, such as Slug, Snail, Twist, ZEB1 and ZEB2, which transform epithelial state into the mesenchymal state [21]. As repored, EMT significantly promoted cancer metastasis, including ovarian cancer, breast cancer and osteosarcoma via some pathways, such as TGF-β, MAPK and NF-κB. It should be noted that EMT also enhanced resistance for radiation and chemotherapy [22]. Thus, drugs targeting EMT biomarkers might be effective and useful approaches for the treatment of cervical cancer patients.

In the present study, we demonstrated BAG3 expression was associated with FIGO stage and metastasis. *In-vitro* analyssi demonstrated that BAG3 siRNAs inhibited the cell growth, invasion and migration. Mechanically, BAG3 siRNAs inhibited the expression of EMT-regulating markers, involving MMP2, Slug and N-cadherin, and increased the expression of E-cadherin. In a xenograft nude model, BAG3 siRNAs could inhibit tumor growth and the expression of EMT biomarkers.

In conclusion, our work suggests that the BAG3 protein can increase the aggressiveness of human cervical cancer. Silencing of BAG3 inhibits the epithelial-mesenchymal transition in human cervical cancer. Thus BAG3 might be recommended as a possible novel way to prevent aggressive growth and metastasis of cervical cancer.

## MATERIALS AND METHODS

### Ethics statement

Ethical approval was obtained from the Institutional Ethics Committee at the Ethics Committee of Shandong Provincial Third Hospital and Shandong Cancer Hospital and Institute. Patients or Animals enrolled in this study signed written informed consent. All procedures were subjected to the Declaration of Helsinki.

### Clinical samples

All clinical samples examined in this study were obtained from surgically removed ovarian tissues of inpatients in Shandong Cancer Hospital and Institute from 2014 to 2016; patients who had received pre-operative radiotherapy or chemotherapy were excluded. 30 patients with cervical cancer were enrolled, including 15 non-metastatic samples and 15 metastatic samples. All of the tumour samples were obtained from the primary tumour site. Diagnosis was confirmed by histopathology in all cases. All protocols were reviewed and approved by the Ethical Committee and all patients gave written informed consent.

The article "Silencing of BAG3 inhibits the epithelial-mesenchymal transition in human cervical cancer" was retracted in 2025. Reasons: plagiarized images; overlap with other authors' work; concerns about the results or conclusions.

### Cell lines and culture conditions

Normal human endocervical epithelial cell (NEEC) was generated from human endocervical samples obtained from biopsies of women (22-23 years of age) who underwent surgery for minor gynecological issues and had no underlying endocervical pathology. None of them had received hormonal therapy in the 3 months preceding sample collection. Samples were minced into fragments <1 mm and subjected to mild collagenase digestion. NEEC was cultured to confluence in a steroid-depleted medium composed of 75% Dulbecco's Modified Eagle Medium and 25% MCDB-105 (Sigma, St. Louis, MO) supplemented with antibiotics, 10% human albumin and 5 mg/mL insulin (Sigma). Human cervical cancer cell lines HeLa and SiHa (American Type Culture Collection) were routinely maintained in DMEM medium supplemented with 10% foetal bovine serum, penicillin (100U/ml), streptomycin (100μg/ml) and amphotericin B (0.25 μg/ml) (Sigma, Poole, UK). Cells were incubated at 37°C with 95% humidity in 5% CO2.

### siRNA transfection

Prior to transfection assay, cells were seeded into 24-well plates with a density of 1 × 105/well. When cells grew up into 80% confluence, siRNA transfection was carried out. 1 mg of control siRNA, or siRNA for BAG3 (target sequence: gcaugccaga aaccacuca), were added to Opti-MEM with Lipofectamine 2000 (Invitrogen) for transfection based on the manufacturer's protocols. 24 hours after incubation, culture medium was changed into fresh DMEM with 10% FBS. Cells were harvested at 72 h following transfection of siRNA. Then cells were subjected to western blotting.

### RNA extraction and reverse transcription PCR

Total cellular RNA was isolated from the CC cells using Tri-Reagent according to the manufacturer's protocol (Sigma-Aldrich, Poole, UK). RNA concentration and quality were determined through spectrophotometric measurement (NanoPhotometer, IMPLEN, Mϋnich, Germany). 500ng RNA was reverse transcribed into cDNA using an Applied Biosystems high capacity reverse transcription kit (Life Technologies, Paisley, UK). DNA quality was verified using GAPDH PCR (sense GGCTGCTTTTAACTCTGGTA; antisense GACTGTGGTCATGAGTCCTT) which was also used as a loading control. BAG3 levels were assessed using primers (sense TCCTGGACAC ATCCCAATTC; antisense TCTCTTCTGT AGCCACACTC). PCR was carried out in an Applied Biosystems thermocycler using a Go Taq green PCR reaction mix (Promega UK, Southampton, UK). Cycling conditions were 94°C for 5 min, followed by 28 cycles of 94°C for 30s, 55°C for 30s, and 72°C for 30s. This was followed by a final 7 min extension period at 72°C. The products were visualized on 2% agarose gel stained with SYBRSafe (Life Technologies, Paisley, UK).

The article "Silencing of BAG3 inhibits the epithelial-mesenchymal transition in human cervical cancer" was retracted in 2025. Reasons: plagiarized images; overlap with other authors' work; concerns about the results or conclusions.

### Western blot analysis

Cell lines were grown to 70% confluence, monolayers were washed with PBS and lysed in ice cold lysis buffer (50mm TRIS, 150mM NaCl, 5mM EGTA, 1% Triton X100 pH7.5) supplemented with protease inhibitor cocktail (Roche, Hertfordshire, UK). Lysates were clarified by centrifugation (12,000 rpm, 15minutes, 4°C) and the protein concentrations in the supernatants were determined using the DC Protein Assay kit (BioRad, Hemel Hempstead, UK). Protein was reduced and denatured by boiling (5min) in Laemmli buffer (Sigma-Aldrich, Poole, UK) and 20μg protein samples were resolved by SDS-PAGE and transferred onto nitrocellulose membrane (GE Healthcare Life Sciences, Buckinghamshire UK). After blocking for 1h in 5% skimmed milk (TBS/Tween: 140mM NaCl; 50mM TRIS, 0.05%Tween pH7.4), blots were incubated overnight at 4°C with primary antibodies Eplin-α (1:500 prepared in TBS/Tween/1% milk) and GAPDH (1:1000 in TBS/Tween/1%milk) (Santa Cruz Biotechnology, Heidelberg, Germany) was used as a loading control. Blots were washed with TBS/Tween and bound antibodies were detected after 1h incubation (room temperature) with appropriate horseradish peroxidase-conjugated secondary antibody (1:1000- Sigma-Aldrich, Poole, UK). Following 3 × 5min TBS/Tween washes, protein bands were visualized using enhanced chemiluminescence (Luminata Forte- Millipore, Herefordshire, UK), and photographed using a UVITech imager (UVITech, Inc., Cambridge, UK).

### Cell proliferation assay

Cells were seeded into 96-well plates at a seeding density of 3,000 cells per well with 12 replicates/experiment. Cells were fixed with 4% formalin after 1, 3 and 5 days growth. Fixed cells were stained with 0.5% crystal violet, washed and dried. Dye was re-solubilised in 200μl acetic acid/well and absorbance was determined at 540nm using an ELx800 multi-plate reader (BioTek UK, Bedfordshire, UK). Each experiment was repeated at least 3 times. For each cell line, analysis compared cell number (absorbance) on day 3 and 5 relative to day 1.

### Cell invasion assay

Cell invasive capability was examined using an *in vitro* Matrigel invasion assay. Transwell inserts (Greiner Bio-One, Stonehouse, UK) with 8.0μm pore size were coated with 50μg Matrigel (BD Biosciences, Oxford, UK), dried at 55°C and rehydrated with 100μl serum-free medium before seeding 4,000 cells per insert. After 48 hours of incubation at 37°C, non-invasive cells and Matrigel were removed from the inside of the inserts with a cotton swab. Cells that had invaded to the underside of the insert were fixed (4% formalin), stained with 0.5% crystal violet and washed. Cell invasion was quantitated by counting the cell number in 4 fields of view (x20 magnification). Data were analysed as mean cell number per field of view for 3 independent experiments with 3 replicates per experiment. Results were confirmed by incubating the stained inserts in 10% acetic acid. Absorbance of solubilized crystal violet was determined at 540 nm.

The article "Silencing of BAG3 inhibits the epithelial-mesenchymal transition in human cervical cancer" was retracted in 2025. Reasons: plagiarized images; overlap with other authors' work; concerns about the results or conclusions.

### Migration assay

A cellular wounding assay was used to study directional cell migration *in vitro* as previously described. In brief, cells were cultured to confluence in a 24 well plate before scratching the cell monolayer with a 10 μl pipette tip. The closure of the induced wound, through the migration of cells, was tracked and recorded over a 36h period using an automated cell imaging system EVOS (Life Technologies, Paisley, UK). Using Image J software, the relative distance cells migrated was calculated using multiple measurements of the width of wound gap after 24 h compared to 0h.

### Tumor xenograft experiments

All experimental procedures were performed in accordance with the National Institutes of Health guide for the care and use of laboratory animals. In all, 1 × 107 cells were resuspended in 100 μl PBS, and injected subcutaneously into the lateral flanks of immunodeficient mice. Tumor volumes were measured weakly, with calculation using the equation: V (cm3) = width2 (cm2) × length (cm)/2. After 4 weeks, tumors were harvested for immunostaining after tumor implantation.

### Statistical analysis

All statistical analysis was performed using the paired t-test for normally distributed data. Differences were considered to be statistically significant at p<0.05.
